The article "Computed Tomography and Magnetic Resonance Imaging Appearances of Abdomen and Pelvis Gossypibomas at the Varied Durations After Cesarean Section" was published in 2021. Journal: Cureus.

# Computed Tomography and Magnetic Resonance Imaging Appearances of Abdomen and Pelvis Gossypibomas at the Varied Durations After Cesarean Section

**DOI:** 10.7759/cureus.18588

**Published:** 2021-10-07

**Authors:** Yu-Feng Bai, Juan-Qin Niu, Chao Zhang, Wen Wang, Jing-Zhong Liu

**Affiliations:** 1 Department of Radiology, The 944th Hospital of Joint Logistics Support Force of People’s Liberation Army, Jiuquan, CHN; 2 Department of Radiology, The 940th Hospital of Joint Logistics Support Force of People’s Liberation Army, Lanzhou, CHN; 3 Department of Radiology, Fourth Military Medical University, Shaanxi, CHN

**Keywords:** diagnosis, magnetic resonance imaging, computed tomography, abdominal, gossypboma

## Abstract

The incidence of gossypiboma is considerably higher in open cavity surgeries, among which cesarean section ranks number one. However, it is difficult to diagnose abdomen or pelvic gossypibomas after cesarean section. We retrospectively analyzed the clinical and imaging data of three pathologically confirmed gossypiboma patients at varied durations after cesarean section. In case one, at four months after cesarean section, a gossypiboma near the small intestine caused fistula and intestinal obstruction. Soft tissue density lesion along the intestinal canal made the “segmental honeycomb sign" and "truncation" with metal markings on the edge on computed tomography (CT). Magnetic sensitivity artifacts were demonstrated as hypointensity on T1 weighted image (T1WI) and T2 weighted image (T2WI), while hyperintensity was seen on the diffusion weighted image (DWI). In case two, a gossypiboma in the peritoneal and intestinal space was revealed with MRI at 18 months after cesarean section. It was featured as a cystic and solid lesion, with "vortex like sign" and obvious ring enhancement on contrast-enhanced MRI scan. In case three, five years after cesarean section, a mass was palpated in the right middle and lower abdomen. MRI revealed a round mass of T1 hypointensity with mixed T2 signal, as well as swirling hypointensity in T2WI, T2WI-fat suppression (FS), and DWI. In CT and MRI examinations for suspected gossypiboma after cesarean section, "honeycomb sign" and "vortex like sign" are the characteristic appearances; gauze translocated into the intestine may show the "truncation sign". Accurate diagnosis is based on the surgery history, symptoms, and imaging features.

## Introduction

A gossypiboma or textiloma is an infrequent complication after any surgical procedure associated with potentially dangerous healthy problems for the patient [1-3] and legal implications for the surgeon [4]. The medicolegal implications and widespread negative press coverage explain why many cases are not reported, with the literature consisting only of case reports [2,3,5]. The incidence of gossypiboma is generally low but is considerably higher in surgeries performed with open cavities, among which cesarean section ranks number one [6]. Early and accurate diagnosis of gossypiboma plays a very important role for delivering proper treatment. However, the diagnosis of gossypiboma is challenging as the symptoms are usually non-specific, may appear years after surgery, and may be misdiagnosed as a tumor [2] or abscess [1,3] in the abdomen and pelvis.

The article "Computed Tomography and Magnetic Resonance Imaging Appearances of Abdomen and Pelvis Gossypibomas at the Varied Durations After Cesarean Section" was published in 2021. Journal: Cureus.

Depending on the retained time of foreign bodies or sponge, exudative, and aseptic fibrous alterations may occur, leading to early abscess or late fistulas [7]. It may also remain clinically silent for many years [8,9]. Thus, radiological imaging is important for accurate diagnosis. Ultrasonography (US) is a cheap and easy imaging modality for gossypiboma diagnosis; however, it may not be sufficient to evaluate the abdominal or pelvic organs in the cases of suspected gossypibomas in women after cesarean section [10]. Thus, recognizing the CT and MRI features of gossypibomas after a varied durations of foreign body retention is very important in this population.

In this study, we retrospectively enrolled three women, who were diagnosed with gossypibomas at varied durations after cesarean section and tried to correlate their imaging features with the pathological findings.

## Case presentation

Case One: Gossypiboma in a woman at four months after cesarean section

A 29-year-old female was admitted to the hospital due to intermittent abdominal pain, abdominal distension, and constipation of gas and feces for more than one month, which got worse in the last two weeks. Intermittent abdominal pain occurred without obvious reason, mainly in the upper abdomen a month ago. The pain became worse after eating, with occasional nausea and vomiting. Recently, she has lost about 15 kg of body weight, which was probably normal after giving birth to a child four months ago. A 10-cm transverse surgical scar was observed at the lower abdomen, together with the whole abdomen tenderness, especially the middle and lower abdomen. Abdomen plain radiograph revealed high density fold line within the lower abdomen (Figure 1A). Coronal reconstruction of plain CT scan revealed tortuous and coiled soft tissue density shadows in the right middle and lower abdominal small intestine, and circular high-density shadows at the edge (Figure 1B). Multiple gas shadows were observed with "segmental honeycomb" changes. Edema and thickening of the intestinal wall and mesentery, dilation, fluid accumulation, and gas accumulation in the upper intestinal layer were also observed (Figure 1B). MRI showed that the fifth group of small intestines occupying the right middle and lower abdomen was dilated, with T2 hypointensity shadows along the intestinal canal lumen (Figures 1C, 1D). T2WI-FS (Figure 1E) and DWI (Figure 1F) hyperintensity and multiple enlarged lymph nodes were observed around the intestine and at the mesenteric roots (Figures 1C-1E). Unfortunately, the corresponding apparent diffusion coefficient (ADC) map was not confirmative (figure not shown). Thus, we did not know whether the water diffusion was restricted within the lesion or not. The patient had symptoms and imaging findings of intestinal obstruction, the bowel is markedly dilated, and laparoscopic surgery was easy to cause collateral injury. Besides, imaging examination showed the thickened mesentery, indicating the peritoneal inflammation. Thus, laparotomy was performed to avoid collateral injury and manage peritoneal inflammatory. During the laparotomy operation, the small intestine was found to have clumps of adhesions at 150 cm from the ileocecal part, and the adhesive bowel was about 40 cm long. An enveloped internal fistula was formed locally. Part of the small intestine was removed, and an enteroenterostomy was performed (Figure 1G). Pathological examination revealed intestinal wall tissue, mucosal tissue degeneration, and necrosis, submucosal vascular dilation, congestion, inflammatory cell infiltration (figure not shown). Based on the patient history and examinations, the diagnosis of intestinal ulcer and perforation with foreign body (gauze) was made.

The article "Computed Tomography and Magnetic Resonance Imaging Appearances of Abdomen and Pelvis Gossypibomas at the Varied Durations After Cesarean Section" was published in 2021. Journal: Cureus.

**Figure 1:** A 29-year-old woman who presented with intestinal obstruction four months after caesarean section. (A) A plain film of kidney-ureter-bladder (KUB) showed a high-density lesion in the hypogastrium (black arrow). (B) Coronal reconstruction of unenhanced CT scan shows honeycombed gauze foreign body in small intestine with visible metal marks (white arrow). (C) Coronal T2WI showed hypointensity lesion along the intestinal canal (white arrow). (D) Axial T1WI showed the isointensity lesion along the intestinal canal (white arrow). (E) Axial T2WI-FS shows a foreign body in small intestine with low signal, and the intestinal wall is swollen and thickened (white arrow). (F) Coronal DWI showed the thickened intestinal wall with the hyperintensity susceptible artifacts at the edge of enlarged lymph node around the intestine (white arrow). Unfortunately, the ADC map for coronal DWI was not available for this case. (G) Postoperative view of the specimen showed a retained surgical gauze foreign body in the mass.

Case Two: Gossypiboma in a woman at 18 months after cesarean section

A 38-year-old female was admitted to the hospital due to intermittent abdominal pain and discomfort for six months. Physical examination showed an old surgical scar in the middle of the lower abdomen, and a soft mass about 8cm×5cm in size was palpable in the left abdomen, with low mobility. She had a caesarean section 18 months ago and had a history of massive bleeding and blood transfusion. MRI examination showed a round 5.5 cm×4.4 cm size mass with hypointensity T1 (Figure 2A) and heterogenous T2 intensity ("swirl-like" sign) (Figure 2B) in the left middle-lower abdomen. The lesion demonstrated uneven hyperintensity on both DWI (Figure 2C) and ADC map (Figure 2D), suggesting non-restricted water diffusion but T2 shine-through effect within the lesion. Besides, a complete hypointensity capsule around the mass can be identified on multi-modal MRI scannings (Figures 2A-2D), which demonstrated as obvious ring enhancement on the enhanced MRI scan (Figure 2E). Laparotomy revealed that the mass in the left middle-lower abdomen was closely adhered to the intestinal canal and mesangium, with a gray-yellow surface. A cystic cavity was visible on the cut surface, and there were pale yellow turbidity fluid and gauze masses in the cavity (Figure 2F). Pathological examination revealed subserosal foreign body (gauze mass), surrounding mesangial and omental tissue, and foreign body granuloma formation in the small intestine (figure not shown).

The article "Computed Tomography and Magnetic Resonance Imaging Appearances of Abdomen and Pelvis Gossypibomas at the Varied Durations After Cesarean Section" was published in 2021. Journal: Cureus.

**Figure 2:** A 38-year-old woman with a mass in her left middle and lower abdomen revealed at 18 months after caesarean section. (A) Axial T1WI showed a round mass with long T1 signal on the left middle-lower abdomen (white arrow). (B) Coronal T2WI showed heterogeneous intensity lesion with a complete hypointensity capsule (white arrow). (C) Axial DWI and (D) ADC showed the hyperintensity lesion (white arrow in C and D). (E) Axial T1 contrast enhanced image revealed ring enhancement of the capsule (white arrow), but without enhancement inside the lesion. (F) Postoperative view of the specimen showed a retained surgical gauze foreign body in the mass.

Case Three: Gossypiboma in a woman at five years after cesarean section

A 30-year-old female with intermittent abdominal pain for two months and abdominal mass for one week was admitted. She underwent cesarean section five years ago, tubal ligation four years ago, and myomectomy one year ago. MRI examination showed a round T1 hypointensity mass (Figure 3A, about 13.1×9.7cm) with mixed T2 signal (Figure 3B) in the right middle and lower abdominal cavity. The “swirling” sign was observed in T2WI (Figure 3B) and T2WI-FS (Figure 3C) images, as well as the heterrogenuous T1 signal (Figure 3A) and hypointensity T2 (Figures 3B, 3C) envelope at the edge of the mass. On DWI, the vortex signal shadow and lower strip band signal can be seen within the hyperintensity background (Figure 3D). However, on the corresponding ADC map, the higher strip band signal was surrounded with hyeperintensity, suggestion metal caused magnetic sensitive artifacts (Figure 3E). On the other layer of DWI (Figure 3F), magnetic sensitivity artifacts can be seen around the high-signal shadow, which was also indicated on the corresponding ADC map as the hypointensity lesion (Figure 3G). Laparotomy revealed a cystic mass at 50 cm away from the ileocecal junction, which encapsulated the ileum and adhered to the adjacent small intestine. The section was cystic, containing yellow fluid and gauze mass, and granulation tissue formation was observed on the cyst wall (figure not shown). Pathological examination confirmed the gauze retention and fibrous tissue wrap, with foreign body granuloma (figure not shown).

The article "Computed Tomography and Magnetic Resonance Imaging Appearances of Abdomen and Pelvis Gossypibomas at the Varied Durations After Cesarean Section" was published in 2021. Journal: Cureus.

**Figure 3:** A 30-year-old woman with a mass in her abdomen revealed at five years after caesarean section. (A) Axial T1WI showed a round hypointensity mass in the right middle and lower abdominal cavity (white arrow). (B) Coronal T2WI and (C) axial T2WI-FS showed heterogenous hyperintensity with a complete hypointensity capsule (white arrows in B and C). (D) Axial DWI showed swirling and hypointensity strip band (black arrow) in the hyperintensity background. (E) Axial ADC showed slight hypointensity and strips of hyperintensity (black arrow) were seen inside. (F) Axial DWI showed the magnetic sensitive artifacts (white arrow). (G) Axial ADC corresponds to F.

## Discussion

Gossypiboma developed after cesarean section is the most common gossypiboma [6]. However, its diagnosis remains a challenge and should be considered in the differential diagnosis of a mass or neoplasm, abscess, lymphocele, or non-specific imaging findings in a postoperative patient [1-3].

Imaging is the most efficient diagnostic approach for gossypiboma after cesarean section. Plain radiography is the most common technique that is easy to diagnose gossypiboma containing a radiopaque marker [8]. Ultrasound (US) may provide sufficient diagnostic evidence in the proper clinical context [10]. However, if the time interval between surgery and symptom onset is prolonged, CT and MRI may have superior advantages to US in differentiating from recurrent tumor, hematoma, or abscess. CT is accurate in diagnosing gossypiboma in the presence of a radiopaque marker or if gas bubbles have developed. Furthermore, some chronic cases of gossypiboma can be identified with the so-called calcified reticulate rind sign, which is probably formed by gradual deposition of calcification along the fiber network of the surgical gauze [11]. However, the gossypiboma with CT for other cases may be more challenging [12]. On MRI, gossypiboma appears as a well-defined mass, showing hypointensity on T1WI and T2WI. The whorl-shaped stripes in the central cavity appear as hypointensity on T2WI [13]. DWI demonstrated some potential in differentiation tumor from cranial gossypiboma in that the later lacks diffusion restriction [14]. This is also true for second case, where the hyperintensity in both DWI and ADC map indicated the T2 shine through effect but not the water diffusion restriction. However, it was not confirmed in case one due to the poor quality of ADC map. It was conspicuous in case three since the ADC map demonstrated higher signal than that of the liver, partially supporting the non-restricted water diffusion within the lesion. Although the locations of gossypiboma were different in the previous (brain) and our study (abdomen and pelvis), it seems that DWI play important role in the differentiating diagnosis of gossypiboma.

The article "Computed Tomography and Magnetic Resonance Imaging Appearances of Abdomen and Pelvis Gossypibomas at the Varied Durations After Cesarean Section" was published in 2021. Journal: Cureus.

In the current study, we presented typical "honeycomb sign" and "vortex like sign" for all three cases of gossypibomas after cesarean section, which is consistent with previous studies showing a spongiform pattern with a radiodense linear structure [11,15,16]. Besides, based on the temporal development and location of gossypiboma, varied imaging features such as cyst, solid soft tissue, or well circumscribed capsulated mass can be observed. These features were not closely related with the disease duration, making the diagnosis of gossypiboma after cesarean section still a clinical challenge. As concluded in previous studies, combining patient history and symptoms with imaging features are important to make the accurate diagnosis.

## Conclusions

If not correctly diagnosed, gossypiboma developed after cesarean section will lead to severe consequences. Imaging plays an important role in accurately diagnosing gossypiboma after cesarean section. The "honeycomb sign," "vortex-like sign," and "truncation sign" on cross-sectional imaging are the characteristic appearances of gossypiboma. Accurate diagnosis is based on the surgery history, symptoms, and imaging features.
